The article "Prospective, randomized evaluation of a personal digital assistant-based research tool in the emergency department" was published in 2008. Journal: BMC Med Inform Decis Mak.

# Prospective, randomized evaluation of a personal digital assistant-based research tool in the emergency department

**DOI:** 10.1186/1472-6947-8-3

**Published:** 2008-01-18

**Authors:** Morris L Rivera, Jason Donnelly, Blair A Parry, Anthony Dinizio, Charles L Johnson, Jeffrey A Kline, Christopher Kabrhel

**Affiliations:** 1 Dept. of Emergency Medicine, Hilo Medical Center, Hilo, HI, USA; 2 Dept. of Emergency Services, Massachusetts General Hospital, Boston, MA, USA; 3 BreathQuant Medical Systems Inc, Charlotte, NC, USA; 4 Dept. of Emergency Medicine, Carolinas Medical Center, Charlotte, NC, USA

## Abstract

**Background:**

Personal digital assistants (PDA) offer putative advantages over paper for collecting research data. However, there are no data prospectively comparing PDA and paper in the emergency department. The aim of this study was to prospectively compare the performance of PDA and paper enrollment instruments with respect to time required and errors generated.

**Methods:**

We randomized consecutive patients enrolled in an ongoing prospective study to having their data recorded either on a PDA or a paper data collection instrument. For each method, we recorded the total time required for enrollment, and the time required for manual transcription (paper) onto a computer database. We compared data error rates by examining missing data, nonsensical data, and errors made during the transcription of paper forms. Statistical comparisons were performed by Kruskal-Wallis and Poisson regression analyses for time and errors, respectively.

**Results:**

We enrolled 68 patients (37 PDA, 31 paper). Two of 31 paper forms were not available for analysis. Total data gathering times, inclusive of transcription, were significantly less for PDA (6:13 min per patient) compared to paper (9:12 min per patient; p < 0.001). There were a total of 0.9 missing and nonsense errors per paper form compared to 0.2 errors per PDA form (p < 0.001). An additional 0.7 errors per paper form were generated during transcription. In total, there were 1.6 errors per paper form and 0.2 errors per PDA form (p < 0.001).

**Conclusion:**

Using a PDA-based data collection instrument for clinical research reduces the time required for data gathering and significantly improves data integrity.

## Background

Since their introduction nearly two decades ago, personal digital assistants (PDA) have secured a place in the pockets of many physicians' white coats [1-4]. The ability to store and conveniently display drug databases and clinical texts garnered early popularity for these devices. Contemporary PDA models are sophisticated computing tools capable of running complex applications such as patient trackers and customizable databases for clinical research.

Researchers have reported changing from paper data collection instruments to PDAs to improve accuracy, efficiency and to reduce the time required to transcribe data from paper to computer databases. Results have been mixed. Some studies report decreased transcription times and improved data integrity [5,6], while other studies highlight shortcomings associated with PDAs such as limited battery life, data loss and cumbersome user interfaces [7].

However, no previous studies have prospectively compared PDA and paper data collection instruments in the emergency department in terms of efficiency, time required, and data errors generated. To address this deficiency, we developed a PDA-based patient enrollment system for an ongoing clinical research study. We compared the collection of research data using paper and PDA forms, examined the time required for data gathering and the frequency and type of errors generated.

## Methods

### Study setting and population

We conducted a prospective, randomized trial comparing two methods of collecting clinical research data: 1. A traditional paper form and 2. A PDA-based data-collection instrument. We compared the two methods in terms of time required for information gathering, the time required for the transfer of data to a computer database, and the number of data errors generated during data collection and/or transcription.

The study was performed from September 2005 until January 2006 in the emergency department of Massachusetts General Hospital, an urban teaching hospital with an annual emergency department volume of 78,000 patient visits. This study was a sub-study of an NIH-funded, prospective multicenter observational study of pulmonary embolism. Patients were eligible for enrollment in this study if they presented to the emergency department and underwent diagnostic testing for acute pulmonary embolism (d-dimer, contrast enhanced computed tomography of the chest, ventilation perfusion scan). Both studies were approved by the human research committee of Partners Health Care. For the sub-study, permission was extended to include the study investigators as study subjects.

### Development of the PDA data collection instrument

We developed a PDA-based version of the research data collection form using the HandDbase™ v3.0 (DDH software, Wellington, FL) application on a Microsoft Windows™ (Microsoft Corp., Redmond, WA) platform. Variables were defined and distributed among ten screen images labeled by numbered tags (Fig. 1). The method of data entry varied according to variable type: check boxes and drop-down menus were used for entering categorical and continuous variables with limited ranges (e.g. temperature, height) while alphanumerical values were entered using the PDA keyboard.

**Figure 1:** **PDA screens**. Ten screen images comprise the PDA form.

Using the CodeWarrior™ Development Studio (Freescale Semiconductor Inc., Austin, TX) for PalmOS™, we developed a "C" program (the "missing data" application) to audit forms and alert the investigator to collect any required data that had not already been entered. Running the "missing data" application required an additional step by the study investigator. We assigned the main database & forms application to one of the main buttons on the PDAs, and we assigned the "missing data" application to another. This simplified the process of checking the completeness of all patient forms resident on a PDA.

Applications were loaded onto four Tungsten-C™ PDAs (Palm Inc., Sunnyvale, CA) running the PalmOS™ v5.0 operating system. All of the PDAs used in this study were password protected. Study PDAs were configured so that study data were uploaded (via "HotSync^®^") from the PDA to a Microsoft Access™ database located on a secure desktop computer.

Programming in Visual Basic 6.0 (Visual Studio 2001, Microsoft Corp.), we created an application to upload data from the Microsoft Access database on the desktop computer to the central study server using a secure SSL network connection with 128-bit cipher strength. Each patient record was transmitted as a single HTTPS POST operation to the study's HTTPS server in the same way desktop browser web forms were submitted to the study server [8].

Investigators already familiar with data collection using the paper form were able to familiarize themselves with data collection using the PDA over a period of about three months prior to initiation of the sub-study. Learning biases associated with use of either instrument were therefore assumed to have been overcome at the time of data collection.

### Patient enrollment and data collection

After informed consent was obtained from patients, but prior to data collection, patients were randomized using a random number generator to have their data collected using either paper forms or PDA. Both the paper and PDA documents used in this study were created for the purpose of the observational research study alone. As such, the study was not intended to impact patient care. Additionally, the data forms did not become part of the patients' permanent medical record.

For each patient who consented to enrollment, we collected data pertaining to patient demographics, past medical history, history of present illness, vital signs, diagnostic and treatment plans as well as the physician's assessment of the pre-test probability for PE. Five study investigators (MR, JD, BAP, AD, CK) enrolled patients. Research data were gathered in a series of two interviews during which an investigator directly queried first the patient's physician and then the patient. Patients were each queried for 62 variables, while their physicians were queried for seven. The remaining variables (patient name, medical record number, social security number and vital signs) were collected in an un-timed step. For a given patient-physician encounter, one investigator gathered all research data. Enrollment was considered complete when all data for a patient were collected.

Patients randomized to paper collection had their data recorded on standard forms. We recorded the time required for study investigators to prospectively collect data from the patient and the physician using a handheld stopwatch. The emergency physician was interviewed first, followed by the patient. Documentation times were reported as the combined times for the physician and patient interviews. Each investigator performed the timing for the patients they enrolled. Times were rounded to the nearest second. Each form was then transcribed by a research assistant onto an e-form located on the study website. A study investigator timed the transcription of each paper form.

Patients randomized to PDA collection had their data recorded directly onto the PDA. Again, investigators recorded the time required to prospectively collect data from the patient and the physician using a handheld stopwatch, with the emergency physician interview being conducted prior to the patient interview. The time required to run the missing-data application was included in timing of the patient interview. Study PDA's were periodically docked onto the desktop computer but the time required to upload ("HotSync^®^") forms from the PDA to the desktop computer and from the desktop computer to the central server was considered negligible.

To determine the rates of data errors using each method, we defined three types of errors a priori: missing, nonsense and transcription. Missing values were those essential entries (e.g. name, telephone number, vital signs) that were not entered. Nonsense values included duplicated entries, atypical values (e.g. numerical values that contained letters, social security numbers of invalid length), impossible vital signs and entries that were illegible to the research assistant transcribing the data. Transcription errors were defined as discrepancies between values entered in the paper form and values on the corresponding e-forms. Error rate determination was performed by a single researcher who manually examined/compared all data collected. The uploading of data from the PDA to the desktop computer was considered to be an error free process.

Sample sizes were powered to detect a difference in data collection times of 60 seconds, using an estimated data collection time of nine minutes for paper (alpha = 0.05, beta = 0.8). Distributions were tested for normality using the Kolmogorov-Smirnov (for error rates) and Shapiro-Wilk (for times) methods. Times were compared using the Kruskal-Wallis equality of populations test for non-parametric values, and error-rates were compared by Poisson regression using STATA 9.1 SE (StataCorp, College Station, TX).

## Results

Our power calculation predicted a need for 21 patients in each study arm in order to detect a difference of 60 seconds in data collection times. Thirty-one patients were enrolled using the paper form, and 37 using the PDA (Fig. 2). Of the 31 paper documents that were completed, 2 were missing at the time of transcription and error-rate determination. As such, total data-gathering times and error-rates could only be reported for 29 paper forms. All of the 37 PDA documents were available.

**Figure 2:** **Study design**. Consecutive patients were randomized to either enrollment instrument. Two paper forms were lost prior to study conclusion.

Mean data collection times were 6:00 minutes for 31 paper and 6:13 minutes for 37 PDA forms (p = 0.460). For the 29 paper forms available at the time of transcription, transcription times ranged from 2:13 minutes to 5:33 minutes per document (mean 3:18 minutes), resulting in a statistically significant difference in mean total data-gathering times between paper (9:12 minutes) and PDA (6:13 minutes). Statistical comparisons for total data gathering times were calculated using matched data-collection and transcription values for each of the 29 available paper forms (i.e. each document's respective data gathering and transcription times were combined).

Error rates were significantly higher for paper (1.6 errors per form) versus PDA (0.2 errors per form; p < 0.001; Fig. 3). Missing data errors occurred most frequently, at rates of 0.8 per paper form and 0.1 per PDA form. Vitals signs accounted for the majority of missing variables for both methods (10/22 for paper; 3/5 for PDA). Nonsense errors occurred at an equal rate of 0.1 per form for both methods. The three nonsense errors found on paper forms resulted from two illegibly written names, and from one uninterpretable response to the question that asked for the period of time that a patient had been post-partum. The four nonsense occurrences on the PDA included three duplicate entries and one mismatched city/state pairing. Transcription generated 0.7 errors per transcribed paper form. Twelve of the 20 transcription errors were in the form of non-transcribed values. The remaining transcription errors were typographical.

**Figure 3:** **Error rates**. Error rates were significantly higher for paper versus PDA.

There were no technical/electrical problems during the study, such as HotSync^® ^malfunction or battery failures.

## Discussion

Clinical studies have traditionally relied on paper and transcription-based data gathering methods that are time-consuming and subject to human error. To address these limitations, investigators have explored the feasibility of using PDAs for data collection.

Early studies showed that PDA-based data collection was limited by short battery life and unreliable memory [7]. However, late model PDAs appear to have remedied these problems, and recent studies have reported reductions in data gathering times and errors as well as improved history-taking and procedural reporting compared to the established paper-based methods. In a cross-over study comparing a PalmOS tool versus a paper and transcription method for collecting clinical data from a computerized patient chart, use of the PDA was associated with a 23% reduction in data-gathering time, measured from the initiation of data collection to the generation of a Microsoft Excel spreadsheet (absolute time difference of 15 minutes per ten forms), as well as a reduction in errors from 6.7% to 2.8% [6]. Another group created a PDA-based collection form for a pain consultation service [5]. Using historical controls, they reported both a reduction in data collection times and improvement in history-taking compared to the established paper-based method [5]. Bird compared emergency medicine resident compliance with self-reporting of procedures using either PDAs or desktop computers, finding no overall difference in effectiveness [9].

There remains a paucity of studies attempting to compare paper and PDA systems in a prospective, randomized manner within the context of a clinical study. We were primarily interested in comparing time and error rate differences as surrogates for efficiency.

Absent a conventional standard, we chose to define a "clinically significant" time difference for data collection to be 60 seconds, a value previously reported in the literature [5]. Despite inherent challenges using the miniaturized PDA screen and keyboard, data gathering times were not significantly different. Importantly, this study was initiated several months subsequent to the development of the PDA program, allowing enrollment personnel to familiarize themselves with the new devices. Hence, it can be inferred that data collection occurred when the learning curve was relatively flat for the use of either paper or PDA instruments.

The ever-present risk of misplacing study data is highlighted by the loss of two paper forms during this study. After study completion, one PDA was lost. It was password protected, and did not contain any study data at the time, but the potential for this problem is worth noting. While PDAs are more expensive to replace than paper, we believe the risk of lost data and patient privacy favor electronic data collection. In addition, wireless networks can be used to securely transfer PDA data from the bedside to a secure database, which can minimize the risk of lost data [10,11].

Missing data appear to have resulted from a combination of human error and features inherent to the data-gathering instrument. The influence of human error was minimized, but not eliminated, by the missing data program we created. Four of the five missing PDA entries occurred on one form, suggesting that (unless the data were simply not available at the time of enrollment) the missing data program was not run. Future endeavors should include efforts to integrate missing data identifiers into database applications. When creating PDA forms parameters may be set to strictly define allowable data values (blank versus essential, letters versus numbers, acceptable ranges) further minimizing the occurrence of nonsense and missing data entries.

Embedded questions (questions that contain sub-variables when certain conditions exist) seem to be particularly prone to incomplete answers. In our study, one embedded question inquired whether the patient had a cough, and if so, asked for the duration of the cough and whether it was associated with sputum production. This question accounted for the greatest number of missing entries among questions that did not require freeform-text entry. For the PDA, this problem was avoided by the creation of drop-down menus that integrated all possible answers into a single response. Others have credited similar improvements in data-gathering to the use of prompt-driven questions, which are felt to more effectively provoke user responses than do blank spaces on paper forms [5].

The potential for observation bias was present owing to the unblinded nature of this study. We did not time the collection of vital signs and certain demographic variables, as these data could be gathered from patient charts, computerized patient records, patients, and unit secretaries. While the time required to gather these data was usually brief, we anticipated the possibility that the transient inaccessibility of any of these sources would require a timely search that would overshadow any differences directly attributable to the enrollment instrument used.

The transcribers used for this study were emergency medicine residents hired at an hourly rate for their services. As such, their lack of formal clerical training may have under-valued the performance of the paper instrument by generating an unusually high transcriptional error rate. On the other hand, our methods were in keeping with our usual practice, which is to use research volunteers to transcribe study documents. Additionally, we did not measure HotSync^® ^times that would serve as a comparison to transcription times. Realistically, the HotSync^® ^step takes a few seconds, during which data from many forms can be collectively transmitted. Therefore, comparing individual transcription times to bulk HotSync^® ^times would have generated no meaningful values. It would have been impractical, and contrary to usual practice, to HotSync^® ^forms individually.

Finally, we did not incorporate into our analysis the time required to program the PDAs or to train the research team in the use of the devices. As such, a broad comparison of resource utilization is limited. However, the forms and systems generated are very flexible once created, and we feel that the initial investment of time is likely to pay for itself over the course of future studies.

## Conclusion

PDAs can be successfully used to collect prospective clinical data in an emergency department setting. PDAs outperform paper-based methods in terms of both efficiency and data integrity.

## Competing interests

The author(s) declare that they have no competing interests.

## Authors' contributions

MLR participated in the design of the study, enrolled patients, carried out statistical analyses, and drafted the manuscript. JD, BAP and AD participated in the design of the study and enrolled patients. CLJ participated in the design of the study, programmed the PDAs and web forms and managed study data. JAK participated in the design of the study, obtained funding, enrolled patients, and participated in drafting the manuscript. CK participated in the design of the study, obtained funding, enrolled patients, and participated in drafting the manuscript

## Pre-publication history

The pre-publication history for this paper can be accessed here:


